# Implementation of a System for Assessing the Quality of Spoken English Pronunciation Based on Cognitive Heuristic Computing

This article has been retracted.

**DOI:** 10.1155/2022/5239375

**Published:** 2022-07-08

**Authors:** Yanping Wu, Changlong Zheng, Meihui Hao, Linlin Wang

**Affiliations:** ^1^Department of Economic Management, Dongchang College of Liaocheng University, Liaocheng, Shandong 252000, China; ^2^Liaocheng Yucai School, Liaocheng, Shandong 252000, China; ^3^Dongchang Middle School of Liaocheng Economic and Technological Development Zone, Liaocheng, Shandong 252000, China

## Abstract

This paper analyzes and investigates the quality assessment of spoken English pronunciation using a cognitive heuristic computing approach and designs a corresponding spoken pronunciation quality assessment system for practical training. Using the general Goodness of Pronunciation assessment algorithm as a benchmark, the shortcomings of the traditional Goodness of Pronunciation method are explored through statistical experiments, and the validity of the overall posterior probability output from the speech model for pronunciation quality assessment is verified. For the analysis of rhythm, there is no common algorithm framework, but in this paper, the *F*0 similarity algorithm based on dynamic time regularization and the stop similarity algorithm based on forced alignment is proposed for the two main factors of rhythm, intonation, and pause, respectively. After framing, the Hamming window processing is used to make the signal smoother, reduce the side lobe size after fast Fourier transform processing, and solve the problem of spectrum leakage. Compared with the ordinary rectangular window function, the Hamming window can obtain a higher quality spectrum. And combined with CTC for speech recognition modeling, the recognition rates are comparable in the case of using BLSTM and bidirectional threshold cyclic unit BGRU as the hidden layer unit, respectively, and the training time is 23% less than BLSTM using BGRU; in addition, the BGRU-CTC model is improved by using a 2-BGRU-CTC model with 256 hidden layer nodes, so that the error rate of phoneme recognition is reduced to 33%. The effectiveness of the algorithm framework is also verified through experiments, which further proves the effectiveness of our proposed phoneme segment feature and rhyme similarity algorithm.

## 1. Introduction

Computer-assisted language teaching (CALL) is an important research direction in the development of speech technology in the field of language teaching, with the main goal of using computers to help language learners better master a second language. Nowadays, increased people need to learn this language, whether it is for further study or in the workplace, and language learning is becoming increasingly important in their lives. The traditional model of learning a second language is to learn a language through teacher instruction and student practice. Real-time instruction and feedback from the teacher often improve the learning process, especially in the case of oral instruction [1]. However, there are some obvious limitations of the traditional teaching model: the number of teachers with the appropriate expertise often cannot meet the huge demand due to many learners; each learner can afford different learning costs (e.g., learning fees); there are time and location constraints in manual teaching, making it difficult for learners to receive immediate feedback and assistance. In this context, computer-assisted language teaching has emerged. In research on computer-assisted instruction for oral language learning, the expectation is that computers can replace teachers or act as aids to teachers, to help second language learners learn a language more effectively [2]. It is easier to be correctly matched; then, the distribution of the posterior probability vector generated by the speaker's speech signal through the acoustic model will generally be more concentrated. In traditional manual instruction, the teacher's largest role consists of standard modeling and real-time feedback and instruction on the student's learning status. While standard modeling can be accomplished by playing a standard model audio recorded by a native speaker, the difficulty and focus of this study are to provide real-time feedback to learners on the standard of their pronunciation, i.e., to assess the quality of spoken pronunciation.

There has been no significant breakthrough in the research on open-ended speaking scoring and assessment techniques. Along with the rise of machine learning technology, some scholars began to study how to apply it to oral language to implement the SpeechRater automatic scoring system with the machine learning compound method. At the same time, researchers in the field also started to provide good ideas for later research, although there is still a gap between the scoring results and teachers' manual scoring. Today, the field of artificial intelligence has undergone new changes, the most significant of which is the maturation of deep learning technology [3]. Deep learning learns data at a deeper level through multilayer networks, uncovering richer features. After many researchers applied this technique to the implementation of speaking score models, the correlation between machine scores and human scores significantly improved and the scoring errors became smaller and smaller. Deep learning techniques have made it possible for open-ended speaking scoring systems to reach a truly practical level.

Many complex systems in the real world can be abstracted as networks composed of entities and the connections between them [4]. The probability value on the corresponding bound state must be significantly larger than the probability value corresponding to other states. Whether it is the social networks initially studied, the gene regulatory networks that control protein expression, or the lexical relational networks of human language, the systemic properties inherent in them are expressed in the form of complex networks. According to the structuralist philosophy, the structure acts as a more essential element than concepts, and in fact, how networks are intrinsically related and how they exhibit diverse structural properties has received more attention from many scholars. Associations, as an intuitive and profound manifestation of the structural properties of complex networks, exist in a wide variety of networks and play an important functional and organizational role. Speech recognition technology has not achieved a certain degree of success in the past, partly because of the backwardness of the technology at that time, and because tools such as the mouse and keyboard can express human commands more accurately than voice. With the increasing maturity of technology, speech recognition has gradually come out of the laboratory and has been applied to people's real life. The classification of speech recognition research can be divided into different tasks according to the needs of different tasks; according to the recognition content, it can be divided into isolated words, connected words, and continuous speech recognition; according to the vocabulary size, it can be divided into small vocabulary, large vocabulary, and very large vocabulary recognition; according to the speaker, it can be divided into the specific person and nonspecific person recognition.

## 2. Related Jobs

By analyzing the articulation patterns and articulatory positions of each phoneme, the phonetic segments of each phoneme are graded according to their GOP values and trained separately, and then, an SVM classifier is trained for each phoneme for articulatory error detection to improve the discriminative ability of the system on articulatory quality [5]. This is the first time that the performance of DBN-HMM is compared with the best-tuned GMM-HMM trained by ML and MWE on the same set of features. Experiments show that the method captures speech errors better than knowledge-based and data-driven speech rules, but at a higher computational cost. DTCWT is used to extract lip texture features because of its displacement invariance and good orientation selectivity [6]. The Canberra distance between adjacent frames of lip texture features is utilized as visual dynamic features. Experimental evaluation of the Chinese corpus shows that visual dynamic texture features outperform static features in visual speech recognition [7]. Compared with the commonly used Canberra distance features, the dynamic texture features can improve the word correct rate by about 8%. In addition, we can also use many data sets for training, which can reduce overfitting while saving the power of the model, but it will make the model learning very computationally expensive. At this stage, Carnegie Mellon University developed Sphinx, an HMM-based speech recognition system that can efficiently perform nonperson-specific continuous speech recognition tasks, and Cambridge University released HTK, which provides a complete set of tools for training and evaluation of speech recognition, and these results have given a great boost to the research of speech recognition technology [8].

In open-ended oral scoring, we need to score the content of the spoken language in addition to the phonological level. The assessment of semantics, vocabulary use, and grammatical accuracy of short texts can be based on ideas from the automatic marking of long texts [9]. Therefore, it is necessary to study “automatic essay correction systems.” Automatic essay scoring is a system for evaluating and scoring essays using techniques from the fields of statistics, natural language processing, and linguistics, and a large body of research has been accumulated in this area. The two models refer to models trained using speech data from native speakers and models trained using speech data from nonnative speakers [10]. The results show that the LLR-based approach performs better than the posterior probability-based approach. However, one problem with this approach is that it requires the use of data from specific nonnative speakers (the target population) for model training [11]. The introduction of background knowledge of the target population's native language can improve the system's pronunciation quality assessment, because by summarizing the observations between the user's first and second language, it is possible to understand the common errors that occur when such first language users learn a second language, thus improving the accuracy of the system [12]. However, it is generally preferred to develop systems that do not rely on knowledge of the first language, which is more conducive to the commercial implementation of the product and avoids a lot of trouble in dealing with languages like Chinese where multiple dialects exist [13].

The correlation coefficient is most consistent with the human sensory evaluation for the comparison of length-regularized fundamental frequency sequences. However, for tasks where the length of the fundamental frequency sequence is an important feature, the mean distance and root mean square distance is more appropriate. However, for the probability distribution whose data space is close to nonlinear manifold data, the modeling efficiency of the Gaussian mixture model is very low. In addition to the length, the range of variation of the fundamental frequency values is also an important influencing factor, because each person's voice conditions are different, and the range of variation of the fundamental frequency values of each person's speech is also different; for example, the range of variation of the fundamental frequency values of women is generally higher overall compared with that of men; if the original extracted fundamental frequency values are directly used for comparison, the comparability of the results will be affected, so it is necessary to do the regularization of the fundamental frequency values of each person. Therefore, it is necessary to regularize the fundamental frequency values of everyone. A deep neural network-based pronunciation quality evaluation algorithm is proposed. The motivation of the proposed algorithm is firstly introduced, and then the outline framework of the algorithm is described, followed by practical applications, and related experimental reports from two perspectives: segmental and rhythmic.

## 3. Analysis of a System for Assessing the Quality of Spoken English Pronunciation with Cognitive Heuristic Computing

### 3.1. English Pronunciation Cognitive Heuristic Computational Algorithm Design

The vowels are pronounced with the lips constantly open, without direct contact with the organs of the mouth, and without obstructing the passage of the articulatory air [14]. The vowels can be distinguished by the roundness of the lips, the position of the tongue, and the degree of tautness of the lips. In the frequency domain, the resonance peaks are the frequency band where the sound energy is concentrated, and there are many other correlations between the resonance peaks and the position of the tongue. There are three resonance peaks for each vowel (*F*1, *F*2, *F*3), and *F*1 and *F*2 are generally used to distinguish vowels. They have their advantages and disadvantages. The earliest method used for resonance peak extraction is the band-pass filter bank method, which has good flexibility in extracting resonance peak features but has poorer performance than the linear prediction method. The inverse spectrum method takes advantage of the small fluctuation amplitude of the spectrum curve to improve the accuracy of the resonance peak parameter estimation but requires high computing power. In contrast, the linear prediction method can simulate a very good vocal tract model, and although it does not match the human ear frequency sensitivity, it is still the most efficient for extracting resonance peaks.

A neural network with one input layer, one output layer, and three hidden layers is usually described with more than 2 hidden layers. Neurons between adjacent layers are connected by weights, and the input *v*^*l*^ and the weights *W*^*l*^ and deviation *b*^*l*^ of the layer are used to obtain the input of the next layer using the activation function.

(1) $$\begin{array}{c} V^{1+1}=f\left(V^{l}W^{l}-b^{l}\right). \end{array}$$

Deep neural nets can be presented in many ways by the different structures of hidden layer units and the different ways of connection between adjacent layers. And for the task of speech recognition, RNNs including their variants have achieved good results and have been widely used.

With sufficient parameters, the hybrid Gaussian model can model probability distributions with arbitrary accuracy requirements to describe arbitrary probability distributions in nature and can be easily adjusted to fit the data using an expectation-maximization algorithm. However, for probability distributions with data spaces close to nonlinear flow-type data, the modeling efficiency of the hybrid Gaussian model is very low. For example, if we need to model a series of points close to the distribution over the surface of a sphere, many Gaussian components are required for a mixed Gaussian model, whereas a very small number of parameters are required if a suitable model is chosen.

(2) $$\begin{array}{c} b_{j}\left(o_{t}\right)=\sum_{m=1}^{M}C_{jm}N\left(O_{t},\mu_{jm},\sum_{jm}\mu_{jm}\right). \end{array}$$

However, its additional hidden layers compared to shallow neural networks allow for better construction of the features of the previous layer, thus allowing for the representation of complex data using fewer dimensions. The most classical deep neural network is the feed-forward neural network, which is trained using the standard back-propagation error derivation algorithm for compartmentalization. The cost function can be determined by the type of learning or the activation function.

(3) $$\begin{array}{c} \Delta W_{ij}\left(t-1\right)=\Delta W_{ij}\left(t\right)-\eta \frac{\partial C}{\partial w_{ij}^{2}}. \end{array}$$

Improvements include weight reduction and stopping learning early, which reduces overfitting but also, potentially, reduces the effectiveness of the model. Alternatively, we can use a large data set for training, which reduces overfitting while preserving the effectiveness of the model, but again, this would make the model learning computationally very large [15]. There are three formants (*F*1, *F*2, *F*3) for each vowel. Generally, *F*1 and *F*2 can be used to distinguish vowels. Thus, a restricted Boltzmann machine-based pretraining process is proposed, which initializes the weight values through the pretraining process, significantly improving the learning of deep neural networks to reduce overfitting and reducing the time to subsequently train the optimized network using the standard error back-propagation algorithm.

For a speaker who is a native English speaker, he is closer to the way of pronunciation in the speech data we use for training the acoustic model and is more likely to be correctly matched than the distribution of the posterior probability vector generated by the acoustic model for that speaker's speech signal will generally be more concentrated, that is, the probability on the binding state corresponding to the intended pronunciation content in the posterior probability vector corresponding to a certain frame. They have their own advantages and disadvantages. The earliest used formant extraction method is the band-pass filter bank method. The band-pass filter bank method has good flexibility in extracting formant features, but the performance is worse than the linear prediction method. The posterior probability vector of a certain frame will be significantly larger than that of other states, as shown in Figure 1.

The posterior probability distribution corresponding to a single frame alone has a great dependence on the specific text information, so the variance analysis is carried out with the posterior probability vector set of only one frame or a small number of frames, which will be largely influenced by the text information. For the same speaker, the larger the amount of speech data selected, the more possible text information is covered, and the effects of different text information on the posterior probability distribution are balanced with each other so that the interference of text information is reduced accordingly and the acoustic information of the sample is highlighted.

(4) $$\begin{array}{c} S_{i}=\frac{M_{i}^{2}}{\sum_{m=1}^{M}d_{m}^{2}}. \end{array}$$

Sound propagation is essentially energy propagation, and the energy loss of high-frequency sound is more serious compared to low-frequency sound. Common mistakes that users of this first language make when learning a second language can be learned, improving the accuracy of the system. Preweighting compensates for the loss of the high-frequency component of the sound and enhances the high-frequency component of it, making the signal smoother in the frequency domain, and the spectrum can be sought by the same signal-to-noise ratio in the complete frequency band. Another point is to remove the response between the vocal folds and the lips during vocalization to highlight the high-frequency resonance peaks.

(5) $$\begin{array}{c} S_{m}^{\prime }=S_{m}+0.95\times S_{m-1}. \end{array}$$

Sound framing is a fixed duration that cut off the sound in the time domain, essentially a fixed number of samples set into a single unit, usually with a value of 512 [16]. Another important aspect is to remove the effect between the vocal folds and the lips during vocalization, which makes the high-frequency resonance peaks more visible. After framing, the audio signal is characterized in units of frames. After frame-splitting, the signal is smoothed by Hamming window processing, which reduces the size of the partials after fast Fourier transform processing and solves the spectral leakage problem. Compared with the normal rectangular window function, the Hamming window can obtain a better-quality spectrum.

(6) $$\begin{array}{c} S_{n}^{\prime \prime }=\left\{0.54+0.46\;\cos\left(\frac{2\pi \left(n-1\right)}{N+1}\right)\right\}*S_{n}^{2}. \end{array}$$

Since the characteristics of the sound signal are better represented in the frequency domain than in the time domain, it is more intuitive to analyze the energy distribution of the sound signal in the frequency domain, and the difference in energy distribution shows the difference in sound characteristics. Therefore, the energy distribution on the spectrum can be obtained by adding windows and a fast Fourier transform. The energy spectrum of the signal can be calculated by squaring and averaging the modulus of the spectrum.

(7) $$\begin{array}{c} P_{k}\left(i\right)=\frac{1}{N}{\left|S_{K}\left(i\right)\right|}_{i}^{2}. \end{array}$$

In this study of automatic pronunciation error detection system, it is necessary to reduce the noise of the input model features as much as possible and include as much information as possible in the learner's pronunciation, to exclude the influence of insufficient features on the error detection accuracy. It can be divided into the recognition of isolated words, connecting words and continuous speech; according to the size of the vocabulary, it can be divided into the recognition of small vocabulary, large vocabulary, and large vocabulary; according to different speakers, it can be divided into specific and nonspecific Identification of a specific person. Among these acoustic features, the resonant peak estimation feature contains less information, and the Meier cepstral coefficient is better than the linear prediction coefficient in terms of signal stability and can maintain good performance when the signal-to-noise ratio is reduced. Therefore, in this paper, the Meier cepstrum coefficients are selected as the feature input for the machine learning algorithm model, as shown in Figure 2.

This part mainly includes dividing the acquired feature data set into training data set and test data set and normalizing them, respectively. The normalization operation does not affect the original distribution of the data. In this paper, a linear function transformation normalization method is chosen.

The signal is first preemphasized using a high-pass filter. Consider that audio signals are quasi-smooth signals. That is, when *N* samples are taken as observation units, they remain relatively smooth and static for a given time of about 15–20 ms, and the time length information of such *N* samples is the framing of the audio signal [17].

However, the frame size should not be too small or too large; otherwise, the spectrum distributed over different time windows on the time axis cannot be obtained. To make a smooth transition between frames, rather than a large variation, an overlapping period can accompany the frames, which is generally taken as one-third of the frame length. In this paper, the sampling frequency of the speech signal is 16 kHz and the frame size is 512 samples, which corresponds to a frame duration of 32 ms and an overlap region of 11 ms.

### 3.2. Design of English Oral Pronunciation Quality Assessment System

Requirement analysis is the first step of the whole system development. This system is designed for English learners to check and correct their English pronunciation problems when they learn English by themselves. The automatic pronunciation error correction system should ensure stable operation. In fact, what kind of internal relationship the network has and how it exhibits diverse structural characteristics have attracted the attention of many scholars. The automatic pronunciation error correction system faces most learners, and to ensure that the learners can check and correct their pronunciation problems without time limitation, the server should be guaranteed to run stably for a long time.

Intelligent oral scoring is a dynamic process from audio input to total score output, and in the scoring system designed in this paper, the process can be described in Figure 3. The candidate's oral recordings are first processed by the speech noise reduction module, and then the speech recognition engine transcribes the clean recordings into the corresponding text content. Then, the data processing module extracts speech-like features and text-like features from the clean recordings and the speech recognition text and inputs the two types of features into the speech scoring model and the text scoring model, respectively. Finally, the output results of the two scoring models are summed to obtain the total score.

In addition to the basic requirements of the system, there is also the main functional business requirement of pronunciation correction. The automatic pronunciation correction system mainly contains two functional modules: the user information management module and the pronunciation correction module. The user management module includes student users, teacher users, and system administrators. The pronunciation error correction module includes the pronunciation data collection module, pronunciation data error detection module, pronunciation data correction module, and historical data display module.

After many researchers applied this technology to the realization of the spoken language scoring model, the correlation between machine scoring and manual scoring has been significantly improved, and the scoring error has become smaller and smaller. While general scoring systems are designed to fit feature values through one scoring model, this paper uses two scoring models (speech scoring model and text scoring model) mainly to improve the accuracy of the scoring system.

In the development process, we adopt the MVC model with the principle of high cohesion and low coupling to develop each functional unit in modules and decouple each module to make the system easy to maintain later and improve the development efficiency [18]. The automatic pronunciation error correction system should be scalable. In the design of a Web system, good scalability is an important aspect of the maturity of the system. The English pronunciation error correction system should be scalable for adding other functions later.

Also, in a real-life grading environment, teachers assess candidates' speaking at the speech and content (text) levels separately. Therefore, such a design is consistent with the manual scoring approach. The design of the core modules in the system will be described in detail later.

Due to the problem of recording equipment, the audio recording often contains current and other noises, which will affect the accuracy of subsequent feature extraction and speech recognition. Therefore, the audio noise is reduced before speech recognition and feature extraction [19]. Traditional noise reduction methods use spectral subtraction or adaptive filtering, but in recent years, due to the successful application of deep learning in the field of speech processing, the use of deep learning techniques in speech noise reduction has achieved very good results and gradually become popular.

This feature is a good indicator of the richness of the spoken content on the one hand and can effectively handle some special data such as empty recordings on the other. The use of words in the text reflects the test taker's vocabulary and proficiency in using the language to some extent, so we extracted the vocabulary richness feature to describe the test taker's use of vocabulary. In the speaking data set used in this paper, the number of words in the text corresponding to each recording is usually around 150, which is a kind of short text without structure, as shown in Figure 4.

The yellow line in each of these box plots represents the location where the median of the data is located, while the upper and lower boundaries of the rectangle represent the location where the upper and lower quartiles are located, so the rectangular area covers the distribution of the modularity values of most of the solutions, and the upper and lower boundaries of the horizontal lines represent the maximum and minimum values in the data distribution.

We can understand this process as the process of human cognition of things around us. People recognize an object not only by its shape but also by combining it with its taste, touch, and other aspects to make judgments. How to provide learners with real-time feedback on the standard level of their pronunciation, that is, oral pronunciation quality assessment, is the difficulty and focus of this research. These features are fused and transmitted to the brain for judgment. In practical applications, feature fusion requires cascading features from multiple modalities after temporal synchronization and then modeling this fused feature by a classifier.

The number and order of video cut frames are important in lip reading prediction because the video frames in the set are arranged in temporal order, and the wrong number or order will affect its performance on dynamic information [20]. After the cut, each frame has a numerical number, and the obtained video frame data set number must be arranged in the order from smallest to largest, without any wrong or missing order; otherwise, it will affect the correspondence of audio and video information in the temporal order.

The feature extraction of audio and video information has been completed in the previous section, but the video stream rate and audio stream are not equally leading to the timing and are not synchronized, if not timing synchronization will lead to the audio information and video information should be the same moment which does not correspond to each other, making the fused features do not have practical significance. Therefore, before feature cascading, the video frame features need to be interpolated to add additional frames between video frames to ensure that the video stream rate is equal to the audio frequency rate. The interpolation process solves the timing asynchronous situation well.

## 4. Analysis of Results

### 4.1. Performance Results of Heuristic Computing Algorithm

Each algorithm was run 100 times independently on each of the six network data sets, and since it was found that the three comparison algorithms were almost guaranteed to converge at 40 iterations during the experiment, the objective function value of the optimal solution obtained at the end of each run (100 iterations) was recorded and counted as the convergence result. The mean, maximum, and standard deviation of the convergence results of 100 runs were calculated at the end of the experiment, and the results are shown in Figure 5.

As can be seen from the experimental results in Figure 5, the EAHAEM-Net method obtains the best results on the maximum value of the objective function and the average value of the objective function after multiple runs on each data set, as well as relatively small deviations, proving the good robustness and high performance of our proposed EAHAEM-Net algorithm. Due to a large number of learners, the number of teachers with corresponding professional skills often cannot meet the huge demand; the learning cost that each learner can bear is not the same; there are time and place limitations in manual teaching, and it is difficult for learners to obtain immediate feedback and help. The reason behind this is that EAHAEM-Net generates high-quality initial solutions not only by sampling operators but also by the physical assumptions behind it; this sampling process can cover a comprehensive division of associations, that is, to maintain the diversity of understanding.

We propose an evolutionary algorithm for community detection based on heuristic sampling and equivalence mapping. It is worth pointing out that although the experiments in this paper use undirected graphs without weights, the two processes, sampling operator and equivalence mapping, are relatively universal, and they solve relatively general problems; for example, the equivalence mapping process can be naturally used in the community detection problems of attribute networks and directed networks, as well as in some combinatorial optimization forms of representation. In addition, the sampling operator plays a significant role in Chapter 4, which helps the evolutionary algorithm to obtain stable association partitioning results from the mapping smoothly, thus enabling effective alternate optimization.

Figure 6 shows the results of the BLSTM-CTC and BGRU-CTC models running with 128 hidden layer nodes and 200 training times. In terms of training time, using GRU as the hidden layer unit is 23% faster than LSTM, while the recognition error rate during the test in the BGRU-CTC model is only 0.36% higher than the BLSTM-CTC error rate, and the two recognition rates are approximately equal.

The time required to train each of the two models is 200 times in each experiment, where the BLSTM-CTC model generally takes more than 4400 seconds to train, while the BGRU-CTC takes less than 3600 seconds on average. GRU has one less gate compared to the LSTM structure and the computational speed is greatly improved. The loss value of the BGRU-CTC model converges before the BLSTM-CTC model as the number of training times increases, and the loss value of the BGRU-CTC model starts to stabilize and stop decreasing at 150 training times, while the BLSTM-CTC model starts to converge at almost 200 training times.

If the language model is removed, the 2-BGRU-CTC model performs better than the above model in theory. In conclusion, an error rate of 33.08% is already a good performance in the current conditions.

The reason for using splicing is that the distribution of the posterior probabilities of different phonemes is closely related to the phonemes themselves, i.e., the textual information, but in the task of this experiment, we expect to learn the information related to the degree of pronunciation in the posterior probability distribution, i.e., the difference in pronunciation between native and nonnative speakers, rather than the corresponding textual information or other interference information. Therefore, adding a reference to the posterior probability distribution of standard recordings can constitute an attention mechanism, which provides the standard posterior probability distribution at the same time as the posterior probability distribution of the input samples each time.

### 4.2. Analysis of the Application of English Spoken Pronunciation Quality Assessment System

After the final score is calculated, the result can be returned to the user. Of course, the purpose of online speaking learning is to make the user's speaking level improve continuously, only giving a score to the user who does not know where their pronunciation errors are, so a method needs to be used to let the user know which words they mispronounce, then continue to train for their mistakes, and finally get the speaking level improved.

By comparing the mismatched points in the two equal sequences, we can get the four mismatched points 6, 7, 8, and 10 and then the correspondence between the template word sequence and the template phoneme sequence. After getting the words that are not pronounced correctly, the user's score is returned and displayed on the interface, and then the user can find out the problems and strengthen the training to standardize their spoken pronunciation, as shown in Figure 7.

To verify the effectiveness of our proposed GAE-EA algorithm on embedding learning, a node classification task is used to compare the quality of the network embedding vectors. Specifically, the network embedding learning algorithm is first executed on the input network topology information, i.e., the GAE-EA algorithm proposed in this chapter and the embedding learning algorithm compared with it, and the result of learning is that each node obtains a feature representation vector. Moreover, the training time of using BGRU is 23% less than that of BLSTM; in addition, the BGRU-CTC model is improved, and the error rate in phoneme recognition is reduced to 33% by using the 2-BGRU-CTC model with 256 hidden layer nodes. Then, a certain percentage of points are randomly selected as the training set, the remaining points are used as the test set, and finally, linear regression is used to perform the correctness test. The reason for choosing linear regression is that it has the most basic feature capturing capability and thus can truly reflect the degree of retention of valid information in the network embedding vector.

The above experimental results show that there are large differences in the correct recognition rates of the three under the addition of noise. The correct rate of multimodal speech recognition with fused video features is significantly higher than the correct rate of speech recognition under unimodal. The reason can be obtained through analysis. In a noisy environment, the extracted audio features are more complicated and contain too much noise, which is difficult to be recognized accurately, but after incorporating video features, the video features are not affected by noise, so the proposed multimodal speech recognition in the noisy environment is beneficial to the improvement of recognition accuracy, as shown in Figure 8.

The sampling operator is used to complement the method of extracting valid information from the network mapping obtained from the self-encoder to form an association representation, thus constructing an alternatively optimized network embedding algorithm. The experimental results show that the accuracy of the classification task can be largely improved by introducing association similarity in the objective function because the association structure can better capture the category information hidden under the node association. It should be noted that in this paper, overlapping associations are only used to optimize the loss function representation, and more structural properties are revealed to be explored later.

Most existing association detection problems based on evolutionary computation do not formally deal with the problem of two solutions having different representational meanings; i.e., they have different semantic environments. In this paper, we take an alternative approach and give a computational method for equivalence mapping from the perspective of Hemming distance and a greedy algorithm with low running time complexity, which dissipates the problem of encoding differences to some extent and does not introduce excessively.

## 5. Conclusion

In this paper, the assumptions of the label propagation algorithm are extended to understand the development of its associations as a label propagation process governed by significant nodes. It is also applied to two processes, initial solution generation and knowledge extraction from graph self-encoders, where the sampling operator can be found to play a significant role. In this paper, a local search system for the association detection problem is gradually developed through the basic association scoring function concept. As the top priority of the results of the dominant algorithm, the local search operator is a powerful tool to improve the solution quality, but people often do not bother to consider whether the function can be computed or estimated in the local view when designing the objective function. Thus, it can guide the direction of the search. Meanwhile, to solve the problem of an unbalanced distribution of sample data based on the MFCC-RF model, the pronunciation classification error detection model of deep belief network and support vector machine is proposed, the model is validated by using the pronunciation data manually labeled by experts in the corpus, and the results show that the DBN-SVM pronunciation error detection model not only overcomes the sample imbalance problem of MFCC-RF model but also expands the pronunciation classification. The results show that the DBN-SVM pronunciation error detection model not only overcomes the sample imbalance problem of the MFCC-RF model but also expands the range of pronunciation classification. Moreover, the accuracy of pronunciation detection is slightly improved. The results show that the DBN-SVM model not only overcomes the sample balance problem of the MFCC-RF model but also extends the range of pronunciation classification and improves the accuracy of pronunciation detection.

## Figures and Tables

**Figure 1:** Framework of pronunciation cognitive heuristic computing algorithm.

**Figure 2:** Flow chart of MFCCRF-based pronunciation error detection model.

**Figure 3:** System scoring process.

**Figure 4:** Average modularity of the solution set obtained by running multiple initialization methods.

**Figure 5:** Algorithm comparison results.

**Figure 6:** Experimental results of BLSTM-CTC and BGUR-CTC under 128 hidden layer nodes.

**Figure 7:** Comparison chart of recombination operator.

**Figure 8:** Effect of alternate optimization on results.

## Data Availability

No data were used to support this study.
